The article "Research on Medical Big Data Analysis and Disease Prediction Method Based on Artificial Intelligence" was published in 2022. Journal: Comput Math Methods Med.

# Research on Medical Big Data Analysis and Disease Prediction Method Based on Artificial Intelligence

**DOI:** 10.1155/2022/4224287

**Published:** 2022-09-09

**Authors:** Fang Zhang, Zhen Zhang, Hui Xiao

**Affiliations:** Information Center, Zhongnan Hospital of Wuhan University, Hubei, Wuhan 430071, China

## Abstract

In recent years, the continuous development of big data, cloud services, Internet+, artificial intelligence, and other technologies has accelerated the improvement of data communication services in the traditional pharmaceutical industry. It plays a leading role in the development of my country's pharmaceutical industry, deepening the reform of the health system, improving the efficiency and quality of medical services, and developing new technologies. In this context, we make the following research and draw the following conclusions: (1) the scale of my country's medical big data market is constantly increasing, and the global medical big data market is also increasing. Compared with the global medical big data market, China's medical big data has grown at a faster rate. From the initial 10.33% in 2015, the proportion has reached 38.7% after 7 years, and the proportion has increased by 28.37%. (2) Generally speaking, urine is mainly slightly acidic, that is, the pH is around 6.0, the normal range is 5.0 to 7.0, and there are also neutral or slightly alkaline. 8 and 7.5 are generally people with some physical problems. In recent years, the pharmaceutical industry has continuously developed technologies such as big data, cloud computing, Internet+, and artificial intelligence by improving data transmission services. As an important strategic resource of the country, the generation of great medical skills and great information is of great significance to the development of my country's pharmaceutical industry and the deepening of the reform of the national medical system. Improve the efficiency and level of medical services, and establish forms and services. Accelerate economic growth. In this sense, we set out to explore.

## 1. Introduction

There is a growing need for an in-depth investigation of the application of logic in artificial intelligence and computer science. The Manual of Logic in Artificial Intelligence and Logic Programming and its companion The Manual of Logic in Computer Science were created to meet this need. A combination of comprehensive investigation and basic research explores underlying topics in various fields. We assume some mathematical complexity as background. Logicians and mathematicians will be interested in most of the material [1]. Constraint programming is currently successfully applied in many areas such as scheduling planning, vehicle routing, configuration, networking, and bioinformatics. But these necessarily focus on the main concepts and technologies and cannot cover extensions, applications, and languages at the same time. The handbook provides a fairly complete coverage of all this work based on constraint programming so that the reader can get a fairly accurate picture of the entire field and its potential. Of course, each work is handled in a survey-like fashion, where some details may be omitted in favor of coverage [2]. Program computation guide artificial intelligence systems Michael Negnievitsky almost all literature on artificial intelligence is in the field of computer science, full of complex matrix algebra, and differential equations. The field of computational intelligence is presented, which includes rule-based expert systems, fuzzy expert systems, frame-based expert systems, artificial neural networks, evolutionary computing, hybrid intelligent systems, knowledge engineering, and data mining [3]. Among various uncertainties, randomness and ambiguity are the most important and fundamental. The relationship between randomness and ambiguity is discussed. Uncertain states and their changes can be measured by entropy and hyperentropy, respectively. The uncertainties of various evolutions and differentiations of chaotic, fractal, and complex networks are studied. A simple and effective method is proposed to simulate uncertainty through knowledge representation, which provides a basis for the automation of logical thinking and image thinking with uncertainty [4]. It is not clear when to monitor the implementation. There is room for improvement, but if the data processing algorithm works, we can use the data processing algorithm outside the original algorithm. So, we cannot use it [5]. Large-scale medical data is a kind of data with large volume, rapid growth, complex structure, and high delay. Write big data machine learning technology applications and medical research progress, including regression analysis, decision trees, subtraction algorithms, low-level machine learning based on basic algorithms, neural network model analysis, and algorithms in big data analysis [6]. The number of outpatient visits in my country has increased significantly, which reduces outpatient time and improves the efficiency of outpatient care. A complementary model based on machine learning is proposed to support diagnosis of outpatients. Other diagnostic models use auxiliary vector machines (SVMs) and neural networks (NNs) to simultaneously classify hyperlipidemia based on clinical features obtained from a set of medical data. The results showed that the diagnostic model was 90% accurate in diagnosing hyperlipidemia [7]. Possible ways to monitor and analyze health conditions is through deep learning algorithms in collaboration with IoT-based medical big data. Recent research trends in related fields usually use traditional machine learning-based algorithms, which are not suitable for IoT-based big medical data due to manual feature extraction and low accuracy. IoT system for health monitoring based on deep learning helps to provide relevant results for different remote doctors in the field of IoT architecture to ensure the understanding of critically ill patients [8]. In the medical field, for the purpose of realizing personalized medicine, innovation has developed from the dissemination of electronic medical records to the accumulation of medical information to the integration of genomic information. However, there is a limit to the manual processing of these accumulated large amounts of information, so it is considered necessary to utilize technologies for medical big data that can be processed effectively and efficiently. Therefore, Fujitsu has developed medical big data analysis technology [9]. The rapid growth of medical data generated by hospital information systems marks the arrival of the era of big data in the medical field. This data has significant value for workflow management, patient care and treatment, scientific research, and education in the healthcare industry. However, the complex, distributed, and highly interdisciplinary nature of medical data highlights the limitations of traditional data analysis capabilities in terms of data access, storage, processing, analysis, distribution, and sharing [10]. The main advantage of the classification system is that, according to the rules of mining associations, they can evaluate multiple tasks at the same time. Association classifiers are especially useful in programs where models help domain experts make decisions. A support system is proposed to predict cardiovascular disease in the Andhra Pradesh population. Experiments show that the accuracy of this set of rules is better than the current system [11]. A systematic review of biomonitoring models can predict the occurrence of disease events in selected drugs. We define pathological events as biological events of interest. These phenomena are characterized as infectious and pathological conditions. We looked at models that try to predict the prevalence of the disease, not just the dynamics of its spread, and models that refer to the national registry of selected factors are of interest in the United States [12]. The medical diagnosis process can be interpreted as a decision-making process in which a physician makes a diagnosis in a new, unknown case based on available medical knowledge and clinical experience. This process can be computerized to present medical diagnoses wisely, objectively, accurately, and efficiently. In recent decades, many researchers have worked to develop effective methods for predicting cardiovascular disease and decision-making systems. Accurate predictions are paramount in these systems [13]. Recent advances in genotyping techniques have allowed the use of large-scale genetic information to identify loci vulnerabilities, a successful discovery that has greatly improved our understanding of complex diseases. Despite these advances, the finding that most genetic effects are minimal for many complex diseases is a major hurdle in developing prognostic models of disease. We compare their accuracy by adapting to different complex diseases. Our results show that penalized regression is generally more stable than current methods and provides better accuracy, at least for the diseases in question [14]. Data mining is the process of extracting useful information from massive data. Data mining has broad application prospects in the medical field. Many researchers have proposed the use of *K*-nearest neighbors (KNN) algorithm for diabetes disease prediction. A different approach has been proposed by some researchers, using *K*-means clustering for preprocessing followed by KNN for classification. These methods result in poor classification accuracy or prediction. For a given dataset, we successfully achieve better results than existing methods. Our second method produces better results than the first method. Classification was performed using a ten-fold cross-validation technique [15]. The second part of the article discusses the application of big data and artificial intelligence technology in medicine. The third part introduces the intelligent model in artificial intelligence. The fourth part predicts the performance of diseases in big data of traditional Chinese medicine and optimizes intelligent methods.

## 2. AI-Based Medical Big Data Analysis

### 2.1. Medical System Application of Artificial Intelligence

#### 2.1.1. Outpatient Registration System

The outpatient registration system is directly related to the current patient consultation process and is also the basis for its construction. The first thing to solve is the registration, which can be processed through the registration app and the medical portal. The outpatient registration system uses JSP technology to realize the intercommunication of related information by completing patient information entry, physician selection, or appointment management. In the process of setting up the system, lay the groundwork for it.

#### 2.1.2. Diagnosis and Treatment System

The diagnosis and treatment system will be operated by physicians, and big data will be constructed based on the machine learning diagnosis and treatment system of big data. In the course of its research, it is analyzed through the collection of existing information, according to the mortality rate, discharge rate, and number of surgeries of existing patients in the hospital. The admission diagnostic criteria are imported; the compliance rate is analyzed; the specific coding value, upper limit value, and threshold value are determined; and then certain control is made. According to the establishment of the diagnosis management system, the existing medical history is analyzed, and then the diagnosis is entered for the patient based on the CT images, MRI, blood routine, and other test results taken by the patient. At the same time, the corresponding diagnosis results are issued to facilitate the continued use of control. And according to the input target to determine the specific standards, in the subsequent use process, do a good job of report analysis and basic maintenance.

#### 2.1.3. Medical Record Management System

The medical record management system is a system that records the detailed information of patients. Based on the automatic concept of machine learning, in the process of model building, the decision tree algorithm is the core, and analysis is made according to the number of evaluations of the existing models. Get the computational status of its kernel model. The establishment of the system will analyze the relevant patient information, the accompanying information of the patient's family, the patient's own medical history, and the patient's disease displacement status. Pay attention to the changing condition of the patient during use and continue to deal with it. This information will be input into the modules in the system, and automatic data generation can also be made according to the input status of the information. The main functions of the preview printing system include the management of daily data, the query of medical records, and the collection of relevant report data. In the maintenance process of dictionary data, medical record function data, and report data, it is managed.

#### 2.1.4. Drug Management System

The drug management system is a kind of system that realizes drug classification as the management core. It integrates big data and can divide drugs into Chinese herbal medicines, western medicines, Chinese patent medicines, etc., realize the printing operation of drug functions, and complete the storage management and control of drugs. In terms of inventory management and preservation and drug functions, in view of the input control characteristics of drugs, medical treatment needs should be combined with big data diagnosis. During the establishment of the drug system, the management of warehousing, taking-out, loss reporting, inventory management, and drug application management is carried out. It is shown in Figure 1.

### 2.2. Current Shortcomings of Medical Big Data

#### 2.2.1. Problems in Data Analysis and Modeling

Health information systems are generally not designed for data research and analysis. In terms of data analysis, medical data is often complex, and the modeling of medical data is closely related to medical business processes, requiring not only professional knowledge in various fields but also genetic experts. That is not possible at that dealership. In other words, how to coordinate experts in different fields to create an effective data model is very important.

#### 2.2.2. Medical Natural Language Processing Is Difficult and Affects Data Quality

Because a lot of detailed patient data is stored in text, the data described in the text is often ambiguous, and there are many specific descriptions of how this structured data is transformed into coherent data: structured data is an important clinical dimensional data processing. One solution is to use natural language. Converting unstructured medical information to structured data requires many forms of medical natural language processing, such as identifying nominal medical topics, nominal auto coding of nominal objects, identifying language search variations of nominal objects, and retrieving temporal information, take data recovery as the core technology.

#### 2.2.3. Poor Quality of Medical Records

Before data can be collected from a research server hub, it must be organized and standardized. This information is required on a case-by-case basis. Base units, time signals, and case data are organized and stored in open standard architectures such as HL7 and CDA to ensure availability and scalability. Offers flexible information retrieval options to help you find the right case. The print interface exports data in standard data formats that third-party platforms can handle. Clinical trials put forward higher requirements on the quality of medical records, and the poor quality of patient data directly leads to differences in clinical trial results, resulting in the precision and validation of data required to write medical records and the standardization of the meaning of each data.

#### 2.2.4. The Compliance of Patients to Provide Follow-Up Data Needs to Be Improved

The follow-up implications of these data for medical research are obvious. During the internship, we learned that most patients with cardiovascular disease are elderly people, and the elderly do not know how to use electronic devices, which affects the speed and accuracy of data collection. In the future, wearables, teleconsultation, and integrity of information systems should be used in healthcare settings in different locations to improve access to healthcare, especially with patients from other countries.

### 2.3. Solutions to the Deficiencies of Medical Big Data

#### 2.3.1. Improve the Efficiency of Doctor Visits

Data visualization can help clients, especially inexperienced clients, to conduct more targeted consultations, as some patients may have errors in their communication and descriptions with clients, resulting in differences in diagnosis and treatment. Systematic visualization of data analysis ensures perfect correlation, even as it helps clinicians learn more. Contact with doctors, especially with patients, becomes more practical and prevents diagnostic errors.

#### 2.3.2. Improve the Quality and Efficiency of Medical Data

Hospital data is for reporting or clinical research purposes only. Due to inaccurate basic medical data standards and high data quality, the query efficiency of traditional database methods is low. Different types of medical data are processed and managed through the medical big data platform and processed through technical means such as word segmentation, structuring, and normalization to improve the quality of medical information. When viewing medical data, a clearer visual interface can be provided. Card checks by hospital staff increase the efficiency of medical information use from 10% to 30% to 80%. This means a significant increase in efficiency.

#### 2.3.3. Improve Hospital Informatization Construction

Hospitals have to deal with standard information items. During the construction of the big data platform, medical data is integrated and processed, data visualization applications are developed, and decision-making, diagnosis and treatment support, and scientific support are provided for hospitals. Hospital data provide rvrf for academic research. It is shown in Figure 2.

## 3. Artificial Intelligence Computing Algorithms

### 3.1. Quantized Convolution Calculation

The quantized convolution calculation is a convolution calculation using the quantized low-bit value, and the quantized convolution calculation that does not require an inverse quantization operation will be introduced. Different from the numerical compression network that needs to perform inverse quantization operation during model inference, quantized convolution calculation only needs to perform sparse prediction (whether it is zero) and does not require inverse quantization operation to restore numerical accuracy, so less computation is required. The amount and less computational complexity, the operation is faster. Formula (1) shows a classical convolution calculation process:

(1) $$\begin{array}{c} Y=\overset{N}{\underset{i}{\sum }}w_{i}⊗x_{i}, \end{array}$$

where the multiplication sign represents the convolution operation. For simplicity of description, the bias is ignored here. For a given quantization function *f*, the corresponding quantization convolution calculation process is shown in formula (2), where the plus sign represents the low-bit numerical quantization convolution operation.

(2) $$\begin{array}{c} f\left(Y\right)=f\left(\overset{N}{\underset{i}{\sum }}w_{i}⊗x_{i}\right), \end{array}$$

(3) $$\begin{array}{c} f\left(Y\right)=f\overset{N}{\underset{i}{\sum }}f\left(w_{i}⊗x_{i}\right). \end{array}$$

Since SeerNet only needs to predict the sparsity of the feature, that is, the spatial position of the zero value in the feature map after the ReLU layer and the max pooling layer, SeerNet does not need to perform inverse quantization. The quantization convolution calculation process is shown in the following formula:

(4) $$\begin{array}{c} \mathrm{sign}\left(f\left(Y\right)\right)=\mathrm{sign}\left(\overset{N}{\underset{i}{\sum }}\left(f_{w}\left(w_{i}\right)⊕f_{x}\left(X_{i}\right)\right.\right). \end{array}$$

In many commonly used CNN models, Conv layers are usually followed by different combinations of batch normalization layers, ReLU layers, and max pooling layers. ReLU makes negative-valued features become zero-valued features, and the max pooling layer allows only one value with the largest absolute value in a subregion to be retained, and all other positions are discarded. Using the quantization network to predict the feature map sparsity after ReLU layer and max pooling layer can save more unnecessary computation compared to predicting only the feature map sparsity after ReLU layer. Depending on how the model experts design the model, the Conv layer, BatchNorm layer, and ReLU layer, the combination of max pooling layers is also different. Since the BatchNorm layer has the greatest impact on feature sparse prediction, SeerNet divides all combinations into the following two types with or without the BatchNorm layer:

(5) $$\begin{array}{c} B=\frac{\alpha \times \left(Y-\mu \right)}{\sqrt{\sigma^{2}+\varepsilon }}+\beta , \end{array}$$

(6) $$\begin{array}{c} B=\frac{\alpha \times \left(\sum_{i}^{N}W_{I}⊗X_{i}+bia-\mu \right)}{\sqrt{\sigma^{2}+\varepsilon }}+\beta . \end{array}$$

By fusing the Conv layer and the BatchNorm layer, SeerNet reduces the computational burden and eliminates the accumulation of quantization errors. Kernel fusion is a common method to accelerate inference of DNN models.

(7) $$\begin{array}{c} f\left(B\right)=f\left(\frac{\sum_{i}^{N}\alpha W_{I}⊗X_{i}+\alpha \times \left(\text{bias}-\mu \right)}{\sqrt{\sigma^{2}+\varepsilon }}+\beta \right). \end{array}$$

### 3.2. Algorithms for AI Computing

By sorting and examining this content, we can deepen our understanding of particle filtration algorithms and their artificial intelligence algorithms and their shortcomings, providing a good basis for further research and refinement of algorithms and to improve future research.

Improve the basic theoretical knowledge of artificial intelligence algorithms, and analyze the adaptive adjustment method at the same time. Through the sorting and learning of these contents, we can deepen the understanding of particle filter algorithm and artificial intelligence algorithm and understand their respective deficiencies, lay a good foundation for subsequent research and algorithm improvement, and improve the efficiency of subsequent research.

(8) $$\begin{array}{c} p\left(x\left|z\right.\right)=\frac{p\left(x\left|z\right.\right)p\left(x\right)}{p\left(z\right)}. \end{array}$$

Using the posterior probability density function from the current moment to the next moment, the system model is used to predict, and the equation used for the prediction is as follows:

(9) $$\begin{array}{c} p\left(x_{k}\left|z_{k}\right.\right)=\frac{p\left(z_{k}\left|x_{k}\right.\right)p\left(x_{k}\left|z_{k}\right.\right)}{\int p\left(z_{k}\left|x_{k}\right.\right)p\left(x_{k}\left|z_{k}\right.\right){dx}_{k}}. \end{array}$$

Let *D* be a random region in *N*-dimensional space, and let *i* be a multiple integral, expressed as

(10) $$\begin{array}{c} I=\int_{D}G\left(x\right)dx. \end{array}$$

Then, its arithmetic mean is

(11) $$\begin{array}{c} g_{m}=\frac{1}{m}\overset{m}{\underset{i=1}{\sum }}g\left(x_{i}\right). \end{array}$$

If these samples are distributed independently, the expectation is

(12) $$\begin{array}{c} E\left[i\right]=E\left[g\left(x\right)\right]=\frac{1}{m}\overset{m}{\underset{i=1}{\sum }}g\left(x_{i}\right). \end{array}$$

Solve problems with random variables. A series of patterns in interstitial space, such as a segment of “particles,” is an approximate distribution. Aggregation of these particles turns the aggregation problem into an aggregation problem, reducing computational complexity and time. If the particle sample is large, the probability distribution may be overestimated.

It can be seen that the algorithm is the optimal filtering method. In practice, fundamental problems are solved with random variables. A set of spatial samples as “particles” are suitable for estimating the distribution. Adding these particles makes the integration problem more than just a summation problem, which reduces computational complexity and reduces computation time. When the particle sample is large, the posterior probability distribution of the problem can be approximated.

### 3.3. Importance Sampling

Assuming that, a random variable *x* ~ *p*(*x*) is estimated, it is difficult to directly extract the sample value in some cases, so an important density function *q*(*x*) can be used to replace the true distribution, and the expected estimated value is

(13) $$\begin{array}{c} E\left[i\right]=E\left[g\left(x\right)\right]=\frac{1}{m}\overset{m}{\underset{i=1}{\sum }}g\left(x_{i}\right), \end{array}$$

where

(14) $$\begin{array}{c} w\left(x\right)=\frac{p\left(x\right)}{q\left(x\right)}. \end{array}$$

Called the importance weight, the sample points are drawn from the proposed distribution function, and the estimated value can be approximated:

(15) $$\begin{array}{c} E\left\{h\left(x\right)\right\}=\frac{1}{n}\overset{n}{\underset{j=1}{\sum }}h\left(x^{i}\right)w\left(x^{j}\right). \end{array}$$

Then, the posterior probability density is

(16) $$\begin{array}{c} p\left(x_{t}\left|z_{t}\right.\right)\approx \overset{N}{\underset{I=1}{\sum }}w_{t}^{i}\delta \left(x_{t}-x_{t}^{i}\right). \end{array}$$

According to the law of large numbers, when *M* is infinitely close to zero, the calculated posterior probability density can be approximately equal to the true posterior probability density. Therefore, the basic steps of the particle filter algorithm are summarized as follows: (1) initialization, including the initialization of parameters such as variance, simulation step size, number of particles, and evolutionary algebra. (2) Extract the particles. When *t* = 0, randomly select *N* particle points from the importance probability density function to form the initial particle set, and the weights are all 1/*N*. (3) Body weight update. Grain weight is calculated using the latest calibration data. The closer the selected part is to the actual subject, the greater the weight given. Grain weight update formula:

(17) $$\begin{array}{c} w_{t}^{i}=\frac{1}{\left(2{\pi \sigma }^{2}\right)}\exp\left(-\frac{d_{i}^{2}}{2\sigma^{2}}\right). \end{array}$$

Normalized weights, normalized calculation of particle weights:

(18) $$\begin{array}{c} w_{t}^{i}=\frac{w_{t}^{i}}{\sum_{i=1}^{N}w_{t}^{i}}. \end{array}$$

Status output is using a weighted method to determine the current target position of the tracking algorithm:

(19) $$\begin{array}{c} x\approx \overset{N}{\underset{I=1}{\sum }}x_{m}^{i}w_{n}^{i}. \end{array}$$

Tracking performance is still inaccurate at some point. There is room for improvement. However, if the data processing algorithm is running, we can use the data processing algorithm outside the original algorithm, so we cannot use it.

It can be seen from the formula that the standard particle filter algorithm can track the target, but the tracking effect is still inaccurate in some positions. There is room for improvement. After learning the whole process of the standard particle filter algorithm through the above part, you can have a deeper understanding of the particle filter algorithm, and at the same time, you can find the areas where the algorithm steps can be improved and prepare the relevant knowledge for subsequent algorithm improvements. In order to better improve the particle filter algorithm, the defect analysis is carried out to obtain

(20) $$\begin{array}{c} x_{id}\left(t+1\right)=x_{id}\left(t\right)+v_{id}\left(t\right). \end{array}$$

## 4. Research on Medical Big Data Analysis and Disease Prediction Methods Based on Artificial Intelligence

### 4.1. Medical Data Analysis under Artificial Intelligence

With the rapid growth of hospital outpatient business, outpatient diagnosis model based on big data analysis technology has become a research hotspot. Researchers are collecting health information from higher-level hospital information systems (SIS). An analysis of data collected over three years shows that the number of outpatients is in the top five in terms of inpatient care is general surgery, gynecology, pediatrics, and emergency. Laboratory clinical trial production increased by 131%. This advancement in outpatient treatment has resulted in a significant increase in wait times for outpatient appointments, which even affects the normal functioning of hospitals under very difficult conditions. The increase in the number of outpatients has greatly increased the burden on outpatients. At its busiest, the average number of diagnoses per doctor increased from 13.2 to 27.6 times. Therefore, it is essential and cost-effective to develop an outpatient auxiliary diagnosis model to reduce the workload of physicians. The proportion of the number of outpatient departments in the top three hospitals is shown in Figure 3.

From the data in Figure 3, we can see that the number of outpatient clinics in internal medicine, department ranks among the top five in 2019-2021. The number of outpatient clinics in general surgery in 2019 was 16.59% and reached 20.99% in 2021; the department with the least number of outpatient clinics was the emergency department, which was only 6.58% in 2019, and increased to 9.97% in 2021. The market size and growth rate of medical big data from 2015 to 2021 are shown in Table 1.

From the data in Figure 4, we can see that the scale of the medical big data market in 2015-2021 shows a steady upward trend, from the initial 606 million yuan in 2015 to 7.905 billion yuan in 2021. From 28.95% in 2015, it increased to 59.37% after 7 years; the year with the highest growth rate was 68.95% in 2019, and the year with the lowest growth rate was only 28.95% in 2015. 2015-2021 my country and the global medical big data market scale is as shown in Figure 5.

### 4.2. Research on Disease Prediction Methods

Comorbidities usually refer to the development of a disorder caused by another disorder or symptom. For example, if a patient develops pneumonia from measles, new pneumonia may be understood as a comorbidity. Another disease or symptom may be due to the development of a disease, such as B. Patients who are prone to muscle pneumonia and new pneumonia can be understood as comorbidities. The combined disease dataset and prediction dataset are shown in Tables 2 and 3.

Take the patient diagnosis table as an example from Table 2. Compared with the first diagnosis, the second diagnosis of the patient is *D*5 and *D*6, so *D*5 and *D*6 can be used as the patient's first diagnosis for future new diseases *D*1, *D*2, *D*3, and *D*4. Secondary diagnosis and two new disease data of *D*1, *D*2, *D*3, and *D*4 > >*D*5 and *D*1, *D*2, *D*3, and *D*4 > >*D*6 shown in Table 2.

As can be seen from the data in Table 3, if *D*7 is a predictive disease, data for *D*7 is added as a positive sample, and samples from other diseases (such as *D*6) are added as a negative sample. The newly created disease record set is scanned, and the new disease records of severe pneumonia are scanned, and the unique code is used as the positive sample to generate the research function, data for disease prediction. The network size of the disease is shown in Figure 6.

From the data in Figure 6, we can see that 77,640 disease genes were collected from MalaCards, UMLS, and other databases, covering 2,978 diseases and 9,012 genes. After analyzing the network nodes, only the prognosis data of severe pneumonia-related diseases were collected, the network was simplified, and finally, a disease co-occurrence network containing 2708 nodes and 218284 edges was constructed based on disease gene associations. The distribution of SG value in urine test generally predicts the occurrence of disease, and the distribution of SG index and disease occurrence is shown in Figure 7.

The data in Figure 7 show the distribution of SG according to urine specific gravity. The graph also shows that across the entire sample, the highest number of cases is 1,015, followed by 1.01 and finally 1.02. This indicates that many patients with pneumonia have an SG of 1.015. The distribution of each gear of pH value is shown in Figure 8.

From the data in Figure 8, we can understand the distribution of each level of pH value, normal urine is usually slightly acidic, so the pH value is 6.0, the normal range is 5.0 to 7.0, but urine below 5.0 is also neutral or slightly alkaline, and vegetarians over 7.0 are considered abnormal. So pH of 7.5 and 8 may be abnormal values in the body.

## 5. Conclusion

In recent years, technologies such as big data, cloud computing, Internet+, and artificial intelligence have continued to develop. As an important national strategic resource, accelerate the improvement of the data transmission service level of the traditional pharmaceutical industry. Implement and promote the deepening and improvement of the reform of the medical and health care system, improve the efficiency and quality of medical services, develop new formats and services, and accelerate economic growth. AI technology can now look for potential clues in patient cases to support a diagnosis, not only providing diagnostic clues and basics to inexperienced young doctors but also helping those with more knowledge find more cost-effective prevention methods.

## Figures and Tables

**Figure 1:** Medical system application of artificial intelligence.

**Figure 2:** Solutions for medical big data deficiencies.

**Figure 3:** The proportion of the number of outpatient departments in tertiary hospitals.

**Figure 4:** Scale and growth rate of my country's medical big data market from 2015 to 2021.

**Figure 5:** 2015-2021 my country and the global medical big data market scale.

**Figure 6:** Disease network scale.

**Figure 7:** Distribution of SG value in urine test.

**Figure 8:** Distribution of pH indicators and disease occurrence.

**Table 1:** 2015-2021 medical big data market size and growth rate.

Years	Market size (100 million yuan)	Growth rate
2015 year	6.06	28.95%
2016 year	9.4	55.12%
2017 year	13.1	39.36%
2018 year	19	45.04%
2019 year	32.1	68.95%
2020 year	49.6	54.52%
2021 year	79.05	59.37%

**Table 2:** Combined disease datasets.

Features									Label
ID	Disease				*D*1	*D*2	*D*3	*D*4	*D*5
1	*D*1	*D*2	*D*3	*D*4	*D*1	*D*2	*D*3	*D*4	*D*6
2	*D*1	*D*2	*D*5	*D*6	*D*1	*D*2	*D*5	*D*6	*D*7
3	*D*1	*D*5	*D*6	*D*7	*D*1	*D*5	*D*6	*D*7	*D*8
4	*D*1	*D*5	*D*8	*D*9	*D*1	*D*5	*D*6	*D*7	*D*9

**Table 3:** Prediction dataset.

Features				Label 1	Label 2
*D*1	*D*2	*D*3	*D*4	*D*5	0
*D*1	*D*2	*D*3	*D*4	*D*6	0
*D*1	*D*2	*D*5	*D*6	*D*7	1
*D*1	*D*5	*D*6	*D*7	*D*8	0
*D*1	*D*5	*D*6	*D*7	*D*9	0

## Data Availability

The experimental data used to support the findings of this study are available from the corresponding author upon request.
